RETRACTED

# Study on Nano Drug Particles in the Diagnosis and Treatment of Alzheimer's Disease in the Elderly

**DOI:** 10.1155/2022/3335581

**Published:** 2022-09-29

**Authors:** ChangQing Li, Yu Xiang, Yunqian Wang, Ping Li

**Affiliations:** ^1^Department of Laboratory Medicine, Chengdu Eighth People's Hospital (Geriatric Hospital of Chengdu Medical College), Chengdu 610000, Sichuan, China; ^2^Department of Laboratory Medicine, The First Affiliated Hospital of Chongqing Medical University, Chongqing, China

## Abstract

**Objective:**

To study the clinical effect of nano drug particles in the diagnosis and treatment of Alzheimer's disease in the elderly, we promote the research on the treatment of Alzheimer's disease and provide basis.

**Methods:**

80 patients with Alzheimer's disease treated in our hospital from April 2021 to April 2022 were selected as the research objects and were divided into the reference group and the observation group by random number table method. The reference group was given traditional treatment drugs, and the observation group was given nano drug particles. The treatment effect, blood lipid level, cognitive function status, and comprehensive effective rate of the two groups were compared, and the treatment data of the patients were scored by ADL and MMSE scale to understand the intelligence level and daily living ability of the patients.

**Results:**

From the comparison results, it is found that the blood lipid level of the control group was in the normal range. The cognitive function of the control group was also better than that of the reference group. The scores of ADL and MMSE in the control group were higher than those in the reference group. The effective rate of the control group was also higher than that of the reference group; *P* < 0.05, with statistical significance.

**Conclusion:**

In the diagnosis and treatment of Alzheimer's disease in the elderly, nano drug particles have good stability and less toxic and side effects, improve the ability of daily living of patients, and have good clinical treatment effect, which is worthy of clinical application.

## 1. Introduction

As the most populous country, China's elderly population has exceeded 200 million. Senile diseases, especially senile dementia, have become a problem that society must pay attention to. Among senile dementia patients, Alzheimer's disease (AD) patients account for 60% to 80%. Liu said that the elderly are the high-risk group of AD, and the elderly aged over 65 have a higher risk of disease. Patients will show cognitive impairment and other symptoms [1]. Zhu and Tong also said that AD is occult in the early stage and is not easy to be found. After suffering from AD, patients will have poor memory, decreased self-living ability, aphasia, and other conditions, and in serious cases, they will have motor dysfunction, urinary system dysfunction, and neurological dysfunction and then lose self-care ability, affecting normal life [2]. The average survival time of patients with Alzheimer's disease is only about 5 years, which is one of the “four killers” threatening the health of the elderly. Hou et al. believe that the harm caused by AD to patients is mainly divided into two points: one is exhaustion; second is that accidents cause self-injury or injury to others [3]. According to the statistics of China CDC, the number of deaths due to AD increased by 57.8% from 2005 to 2016.

RETRACTED

Cheng et al. said that, in China, there are more than 7 million patients with AD [4]. According to the survey results released by China Alzheimer's Association in 2011, about 36.5 million people worldwide suffer from dementia, and one person suffers from dementia every seven seconds. Wang et al. predicted that, by 2050, the number of AD patients in China may reach 30 million [5]. Yang et al. said that the condition of AD is complex and diverse, which will not only bring great harm to the normal life of patients and their families but also cause a heavy burden on medical institutions and the country [6]. AD has caused serious harm to social health.

Research on the treatment of AD has been ongoing. Zhang et al. said that, after brain tissue examination, AD patients generally have a large number of extracellular neurons in the brain *β*-amyloid protein (*β*-amyloid A *β*) pathological phenomena such as senile plaques (SP) formed by deposition, neurofibrillary tangles (NFTs) formed by abnormal phosphorylation of tau protein, and neurodystrophy [7]. The abnormal tau protein will lose its stabilizing effect on microtubules, cause the functional degradation of nerve cells, and cause the corresponding nervous system diseases. Sun et al. also said that at present, there is no radical cure for AD, and only drug treatment can regulate some neurotransmitters in the brain, so as to reduce symptoms and delay the development of the disease [8]. Oxford et al. said that the traditional oral dosage form is the main treatment medicine used in AD clinic at present, which lacks brain specificity. At the same time, the existence of blood brain barrier (BBB) in the central nervous system prevents drugs from entering the brain, and the drugs have been inactivated before reaching the action target [9].

The treatment of AD is in trouble and more effective treatment strategies are urgently needed. At this time, nano drug particles came into the sight of researchers. Masoudi Asil et al. said that the nano drugs studies include nanoparticles, solid lipid nanoparticles, carbon nanotubes, nano carriers, polymer micelles, antibodies, and their complexes [10]. Zhang et al. said that nano materials have higher safety and effectiveness. Because of its small size, it can easily penetrate the BBB to reach the lesion as a drug delivery carrier and plays an indispensable role in the treatment of AD [11]. The drug substances wrapped by nanoparticles enter the human body and enter the capillaries through blood circulation, improving the bioavailability of drugs. Wang et al. also agreed with nano materials. She said that the nano carrier of nano preparation can effectively penetrate the BBB, improve the bioavailability of drugs, and even achieve targeted transmission.

RETRACTED

This paper mainly studies the clinical effect of nano drug particles in the diagnosis and treatment of elderly patients with AD. The purpose is to provide reference for the research of nano drugs in AD and contribute to the in-depth research in the field of AD disease through the analysis of the clinical effect of nano drug particles.

## 2. Data and Methods

### 2.1. General Information of Patients

80 patients with AD admitted in our hospital from April 2021 to April 2022 were selected as the research objects. They were randomly divided into the reference group and the observation group. One group was given traditional treatment drugs and the other group was given nano drug particles. The reference group consisted of 40 people, 15 men, and 25 women, aged from 60 to 78 years, with an average age of 69.89 ± 2.70 years. There were 40 people in the observation group, 19 men and 21 women, aged from 61 to 80 years, with an average age of 71.53 ± 2.56 years. There was no significant difference in the general data between the two groups, which was comparable.

### 2.2. Case Inclusion Criteria and Exclusion Criteria

#### 2.2.1. Case Inclusion Criteria

1. The patient's family members agreed to support the study;
2. he patient's Age ≥60 years old;
3. he patient was diagnosed with AD by CT, EEG, and other examinations.

#### 2.2.2. Case Exclusion Criteria

1. Quitting the researcher halfway;
2. atients with tumor diseases;
3. atients who have recently undergone surgery.

### 2.3. Observation Indicators

1. The therapeutic effects of the two groups were compared;
2. he cognitive function status of the two groups was compared;
3. bserving and recording the mini mental state examination (MMSE) of patients after treatment;
4. bserving and recording the patient's activity living scale (ADL);
5. bserving and recording the treatment efficiency of the two groups of patients.

RETRACTED

### 2.4. Efficacy Evaluation Criteria

1. Significantly effective: after treatment, the MMSE and ADL scores of patients increased by more than five points, including five points. Patients can complete daily living activities independently.
2. Effective: after treatment, the MMSE and ADL scores of patients increased by more than two points. Although they reacted slowly, they could understand simple questions and answers.
3. Invalid: the improved specified standard score is not reached.

## 3. Method

### 3.1. Treatment Method

The control group was given traditional treatment drugs, cholinesterase inhibitors, glutamate receptor antagonists, and other treatment drugs. The observation group was treated with nano drug particles (inhibit a β drug delivery system of the prepared drug). Both the groups were treated for 45 days.

### 3.2. Statistical Analysis Method

According to the research information obtained by the above method, the IBM SPSS 24.0 platform is used for analysis and management. The measurement data were expressed in ($\bar{x}$ ± *s*), and the counting data were expressed in rate (%), using t-check. In all the analyses, when *p* < 0.05, the statistical results are considered to be statistically significant.

## 4. Simulation Verification

### 4.1. Comparison of Blood Lipid Levels

Abnormal blood lipid levels play a certain role in the pathogenesis of AD. Blood lipids tend to be stable under normal circumstances, but blood lipid levels are also easily affected by disease-related factors. Abnormal blood lipid levels are an important risk factor for the occurrence of AD. The four items of blood lipids include TC, TG, LDL-C, and HDL-C. Now, the blood lipid levels of the two groups are compared and analyzed. According to the data information, Table 1 is obtained.

Table 1 shows the comparison results of blood lipid indicators of patients. The blood lipid level of patients taking nano drug particles is within the normal range, and the blood lipid level of patients taking traditional drugs is a little abnormally high; *p* < 0.05, with statistical significance. The change of blood lipid level in the course of AD patients is an important risk factor for patients.

According to the data information in the above table, Figure 1 is obtained.

As shown in Figure 1, we compare the two groups of information data, and there is a statistical significance of *t* < 10.000, *p* < 0.05. It is obvious that there is a great difference between TC and HDL-C in the two groups of data, which indirectly shows that nano drug particles are ideal for controlling blood lipid indicators and have a certain stabilizing effect on AD patients.

### 4.2. Analysis of Cognitive Function

The age of aging is coming, which makes the incidence rate of AD gradually increase. AD is an irreversible neurodegenerative disease. Memory loss is one of the most common early symptoms of AD and the most common and prominent symptom in the early stage of the disease. In daily life, sports behavior is difficult, language expression ability and understanding ability will be declined, it will be difficult to accurately judge things, and there will be feeling of extreme difficulty when accepting new things and obvious cognitive dysfunction. According to the statistical results of the two groups of patients, Table 2 is obtained.

RETRACTED

Table 2 shows the analysis results of memory function, motor behavior function, and language expression function of AD patients. The data results of patients with nano drug particles are about 85%, and the cognitive function is significantly better than that in the reference group.

According to the statistical results in the above table, Figure 2 is obtained.

As shown in Figure 2, compared with the different drug effects of the two groups, nano drug particles can effectively improve the morphological changes of neurons in patients, save the memory impairment of patients, and delay the onset process.

### 4.3. Comparison of the ADL Score and MMSE Score

AD patients take nanoparticle drugs. When the nanoparticles reach the inflammatory area of the brain, the chemical reaction caused by them can eliminate the proinflammatory cells and reduce the level of inflammatory factors. At the same time, nanoparticle drugs have the dual functions of diagnosis and treatment. In this study, the two groups of patients were given the ADL score and MMSE score. The ADL score is mainly aimed at the assessment of patients' activities of daily living. The total score is 100 points according to the Bi index. The higher the score, the less dependent the patient is. The MMSE score is a screening of patients' cognitive and intellectual functions. The total score of the result evaluation is 30 points, and a score lower than 27 is considered as cognitive dysfunction. Now, according to the information of the evaluation scale, Table 3 is obtained.

In Table 3, the score value is in direct proportion to the patient's ability of daily living and is also directly related to the patient's intellectual and mental state. The observer uses nano drug particles to improve his intelligence, mental state, and ability of daily living. The treatment effect is ideal, safe, and reliable.

According to the information results of the two groups of evaluation scales, Figures 3 and 4 are obtained.

As shown in Figures 3 and 4, the visualization effect of the ADL and MMSE evaluation results is shown. It can be seen intuitively that the two scores of elderly AD patients in the observation group are higher than those in the reference group, which indirectly shows that nano drug particles can effectively maintain the normal nervous system of patients in the treatment of elderly AD patients, so as to ensure brain nerve function.

RETRACTED

### 4.4. Comparison of Treatment Effectiveness

The disease attacks the brain of AD patients, affects the memory, language ability, and even the most basic thinking process of the elderly, and seriously endangers the health. Nanoparticles can improve the effect of drugs on brain entry efficiency and the accuracy of drug administration, and the antioxidant effect of nanoparticles can effectively remove reactive oxygen species. It can inhibit the atrophy of hippocampus. Now according to the statistics of significant effectiveness, effectiveness, and ineffectiveness, the final comprehensive effective rate is obtained. According to the effective rate of patients, Table 4 is obtained.

Table 4 shows the number of patients with nano drug particles with significant treatment effect has exceeded half, and the number of ineffective people is very small, and the comprehensive effective rate of treatment is as high as 92.5%. The use of this drug can play a more significant effect on AD patients.

According to the visualization of the treatment effectiveness in the above table, Figure 5 is obtained.

As shown in Figure 5, the visualization effect of the treatment is shown. The difference drug treated patients in the treatment effectiveness is not obvious. In the significantly effective treatment, the number of effective patients accounts for a large proportion, and the proportion of the reference group in the treatment ineffectiveness is also very high. The comprehensive effective rate of the two groups of patients has also opened a significant gap, indicating that nano drug particles can effectively control the progress of Alzheimer's disease; it can bring good news and hope to the majority of AD patients.

## 5. Discussion

Nano drug particles can improve the absorption and targeting of drugs in the diagnosis and treatment of AD patients. The structure of nano particles can significantly improve the concentration of drugs in the brain, improve the therapeutic effectiveness of brain tissue diseases and brain nervous system diseases, and reduce the memory impairment of patients. Xiang et al. said that at present, AD has become one of the most serious problems faced by geriatrics. It can effectively control and prevent the cognitive decline of elderly patients with AD and the behavior change caused by the disease [12]. Traditional drug treatment can only alleviate the development of the disease. At the same time, BBB prevents drugs from entering the brain, which makes AD treatment more difficult. The use of nano drug particles can better solve this problem. El-Sayed and Kamel said that nano drugs enhance the penetration ability of BBB and have low invasiveness. At the same time, they can improve the drug transmission capacity [13]. Nano drugs not only improve the therapeutic effect but also reduce the side effects of drugs.

RETRACTED

The clinical treatment of AD patients is to control the disease symptoms, delay disease progression, and improve patients' quality of life, cognitive promotion, rehabilitation, and functional exercise, which can improve the symptoms of AD patients. Highly functional nanoparticles can accurately deliver drugs to AD lesions, with targeting mechanism, pharmacodynamics, and safety. The AD symptoms change over time, and the speed of its progress is also variable. Once the symptoms of the disease appear, recovery has become impossible. After all, brain injury has occurred, so it is urgent to develop effective drugs to treat AD. The clinical effect of nano drug particles is still considerable. However, nano drugs are not without shortcomings. Wong et al. believe that there are differences between nano drugs and traditional drugs, so the safety of nano drugs cannot be evaluated by using the scheme of traditional drugs. At the same time, due to the self-modification of nano drugs, the mode of administration, and the complex structure of brain cells, it is difficult to study the biosafety of nano drugs [14].

In the follow-up of nanotechnology in drug research, a perfect evaluation system should be established to promote the further research and development of nano drugs.

## 6. Summary

With the rapid development of nanotechnology, it has provided new solutions in the field of biomedicine and the treatment of AD patients. In this study, traditional drug therapy and nano drug particles were used to compare the treatment effects in elderly patients with AD. The elderly patients with AD were evaluated by scoring scale, and the patients' ability of daily living and cognitive dysfunction were analyzed and discussed. It can be seen that nano drug particles will improve the blood lipid level of patients, improve the daily living ability of AD patients, and improve the cognitive memory function of AD patients. The treatment obtained by nano drug particles in the treatment of patients in this study has been more effective. Nanotechnology will help promote the clinical application of nano medicine and provide a basis for the further scientific research of AD disease in the future. It has a certain application prospect.

RETRACTED

## Figures and Tables

**Figure 1:** Visualization of blood lipid levels (mmol/l).

**Figure 2:** Visualization of cognitive function (%).

**Figure 3:** Visualization of the ADL score results.

**Figure 4:** Visualization of the MMSE score results.

**Figure 5:** Visualization of treatment effectiveness (%).

**Table 1:** Analysis of blood lipid levels (mmol/L).

Group	TC	TG	LDL-C	HDL-C
Reference group	6.24	1.72	1.55	3.41
Observation group	5.01	1.55	1.35	2.98

**Table 2:** Analysis of cognitive function (%).

Group	Memory function	Motor behavior function	Language expression function
Reference group	67.89	70.53	70.12
Observation group	85.32	84.78	85.08

**Table 3:** Comparison of the ADL scores and MMSE scores.

Group	ADL	MMSE
Reference group	74	24
Observation group	92	29

**Table 4:** Comparison of treatment effectiveness (%).

Group	*n*	Significant effective	Effective	Invalid	Comprehensive effective (%)
Reference group	40	12(30%)	16(40%)	12(30%)	70
Observation group	40	22(55%)	15(37.5%)	3(7.5%)	92.5

## Data Availability

The data underlying the results presented in the study are available within the article.
